# Activated Hepatic Stellate Cells Promote the M1 to M2 Macrophage Transformation and Liver Fibrosis by Elevating the Histone Acetylation Level

This article has been retracted.

**DOI:** 10.1155/2022/9883831

**Published:** 2022-09-12

**Authors:** Junru Chen, Xueqing Huang, Zhi Huang, Yu Cao

**Affiliations:** ^1^Department of Dermatology and Venereology, College of Clinical Medicine, Guizhou Medical University, Guiyang 550025, China; ^2^The Maternal and Child Health Care Hospital of Guizhou Medical University, Guiyang 550003, China; ^3^Department of Intervention, The Affiliated Hospital of Guizhou Medical University, Guiyang 550002, China; ^4^College of Greater Health, Guizhou Medical University, Guiyang 550025, China

## Abstract

Liver fibrosis results from the formation of fibrous scars of hepatic stellate cells by various chronic liver diseases. Considering that the liver is the most important metabolic organ in the human body, exploring the metabolic characteristics of liver fibrosis is expected to discover new markers and therapeutic targets. In this study, we first used mouse model to verify that both lactate content and histone acetylation levels were significantly increased in hepatic fibrosis mice. At the same time, it was confirmed that activated hepatic stellate cells (HSCs) cocultured with M1 macrophages can promote their transformation into M2 macrophages in hepatic stellate cell line and primary hepatic stellate cells. In addition, the addition of lactic acid to the medium in which M1 cells are cultured can promote their transformation into M2 macrophages. Therefore, we concluded that activated HSCs can promote the transformation of M1 to M2 macrophages through lactate accumulation, thereby causing liver fibrosis.

## 1. Introduction

Hepatic fibrosis is characterized by the formation of fibrous scar by the accumulation of extracellular matrix components after liver injury caused by various chronic liver diseases [1]. If not effectively controlled, liver fibrosis can develop into liver cirrhosis and even liver cancer [2]. In fact, cirrhosis is reversible, and effective antifibrotic therapy can significantly change the treatment and prognosis of patients with liver disease [3, 4]. So, it is very important to explore the mechanism of liver fibrosis and find effective methods to inhibit it.

It is generally believed that the activation of hepatic stellate cells (HSCs) is the key cause of the occurrence and development of hepatic fibrosis [5]. In physiological state, HSCs are quiescent [6]. When the liver is injured, quiescent HSCs become activated HSCs by downregulating the expressions of vitamin A and peroxisome proliferator-activated receptor *γ* (PPAR*γ*) [7, 8]. Subsequently, activated HSCs migrate to the liver injury site, secrete extracellular matrix, and form a fibrous scar [9]. Interestingly, recent studies have shown that activated hepatic stellate cells can increase the enrichment of hepatic M2 macrophages, and the number of hepatic M2 macrophages is positively correlated with the severity of liver fibrosis [10]. In fact, as the first line of defense against pathogens, hepatic macrophages are involved in all stages of liver fibrosis, from initiation of inflammation and progression of fibrosis to degradation of fibrous collagen and regression of scarring [11, 12]. M1 and M2 macrophages, the two most typical phenotypes of hepatic macrophages, mediate hepatic inflammation and tissue remodeling, respectively [13]. Interestingly, phenotypic switching between M1 and M2 can occur under specific stimuli in vivo and in vitro [14]. Therefore, it is of great significance to study how M1 and M2 are transformed and their relationship with HSCs for the treatment of liver fibrosis.

The liver is a key metabolic organ that controls energy metabolism in the body, and its life activities produce thousands of metabolic small molecules [15]. These small molecules are not only the products catalyzed by enzymes but also can affect the function of proteins through covalent modification [16]. Recent studies have found that lactate accumulated during metabolism can act as a precursor to lactate modification of histone lysine and participate in the homeostatic regulation of bacterial-infected M1 macrophages [17, 18]. Interestingly, elevated levels of glycolysis are a hallmark of HSC activation [19], and glycolysis can generate large amounts of lactate, which can as a substrate to catalyze lactate modification of histones. Importantly, elevated levels of acetylation in M1 macrophages promote their transformation into M2 macrophages [20]. So, we speculate that activated HSCs can increase the level of histone lactate modification in M1 macrophages by secreting a large amount of lactate, thereby promoting the transformation of hepatic macrophages from M1 type to M2 type and promoting the progression of liver fibrosis. Moreover, histone deacetylase inhibitors (HDAC inhibitors) have also been used as a class of clinical drugs [21]. It is a great pity that there is no effective treatment for liver fibrosis other than liver transplantation. Therefore, revealing the regulatory mechanism of lactate, a metabolite of HSCs, has important scientific significance for understanding the occurrence, diagnosis, and treatment of liver fibrosis.

In our study, we first constructed liver fibrosis mice and examined the changes in lactate and histone acetylation levels in the model mice. Then, we clarified the relationship between HSC activation and macrophage transformation by coculture of HSCs with M1 macrophages. Furthermore, we revealed whether activated HSCs could cause liver fibrosis through lactate accumulation with macrophage transformation. Therefore, the current study may provide a theoretical basis for the therapy of liver fibrosis.

## 2. Materials and Methods

### 2.1. Mouse Treatment and Tissue Section

All the mice used in this study were purchased from Shanghai SLAC Laboratory Animal Co., Ltd. All animal experiments were approved by the institutional animal care and use committee (IACUC) of Guizhou Medical University (approval no. 2101003). 8-week-old female mice were intraperitoneally injected with 1 ml/kg carbon tetrachloride (CCl4; Sigma, in peanut oil) twice a week for 8 weeks before ultrasound imaging was performed to assess liver cirrhosis. Each group contained 12 mice. Animals were sacrificed when the mice were moribund and livers were used for subsequent analysis.

### 2.2. Pathological Examination

The livers were weighed, fixed in 3.7% formaldehyde solution, embedded in paraffin, then sectioned (4 *μ*m) with a paraffin microtome. Paraffin sections were then roasted at 60°C for 2 h, dewaxed in xylene, gradient alcohol rehydrated, and routinely stained by applying hematoxylin and eosin (H&E) staining. And the results were observed and photographed under a light microscopy. The pathologic structure was analyzed by 2 pathologists independently to observe the degree of inflammation and fibrosis of liver tissue. Based on the studies [22, 23], paraffin sections were also routinely processed before performing Masson and Sirius red staining. And the data were observed and photographed under the light microscope.

### 2.3. Cell Culture and Activation

LX-2 cells were cultured in Dulbecco's modified Eagle medium (DMEM; Gibco, Rockville, MD, USA, 21068028) supplemented with 10% fetal bovine serum (FBS; Gibco, 10099141C), 50 U/ml penicillin and 50 *μ*g/ml streptomycin (Gibco) at 37°C in humid incubator containing 5% CO_2_. According to You et al. [24], for activation, LX-2 cells were cultured in DMEM containing 2% FBS and 10 ng/ml transforming growth factor-*β* (TGF-*β*; Cell Signaling Technology, Inc., Danvers, MA, USA, cat. no. 2519) for 48 h. Primary HSCs were isolated from C57BL/6 mice according to the study [25], and TGF-*β* was used for activation of HSCs. M1 macrophage was transformed form THP-1 cell by treating with 100 ng/ml lipopolysaccharide (LPS; Sigma-Aldrich, St Louis, MO, USA) for 12 h. To detect the specific mechanism of transformation from M1 to M2 macrophage, M1 macrophage was treated with 20 mM lactate for 24 h.

### 2.4. Isolation of Primary Mouse HSCs

After the circular perfusion using 0.05% Type IV collagenase (Sigma) and 0.01% Pronase E (Sigma) to remove liver collagen tissue, the HSCs were isolated by density gradient centrifugation. All the cells after digestion were centrifuged in 18% Nycodenz (Sigma) at 3200 rpm for 15 min. Then, HSCs were distributed at the middle layer. Primary HSCs were cultured in DMEM (Gibco) supplemented with 20% FBS at 37°C 5% CO_2_.

### 2.5. Western Blot

Protein extracts were prepared from equal number of cultured cells or equal weight of liver tissue using 1× SDS loading buffer. Equal volumes of protein liquid were separated by SDS-PAGE gel electrophoresis, transferred to polyvinylidene fluoride (PVDF; Millipore, IPVH20200 membranes), and incubated with the anti-Kla (PTM bio), anti-histone H3 (Cell signaling technology, CST4499s), anti-*α*SMA (Abcam, ab32575), or anti-GAPDH (Proteintech, 60004-1-Ig) overnight at 4°C. Blots were visualized with HRP-conjugated secondary antibodies (Jackson, 115-035-003). And the signal was analyzed using the enhanced chemiluminescence reagent (Beyotime, China, P0018FM).

### 2.6. Chromatin Immunoprecipitation (ChIP) Assay

ChIP assay was carried out as the method of Lan et al. [26]. M1 macrophages were crosslinked with 1% formaldehyde for 10 mins and then stopped by 125 mM glycine. After lysis and sonication, 3 *μ*g of Kla (PTM bio) antibody was incubated with chromatin sample overnight at 4°C, and 20 *μ*l protein A/G beads (Smart lifesciences SA032005) were used for immunoprecipitation. Finally, DNA were purified with PCR recovery kit (QIAGEN #28006) and used for qPCR analysis. And the protein sample was analyzed by western blot to detect the histone acetylation level.

### 2.7. Reverse Transcription Quantitative Polymerase Chain Reaction (RT-qPCR)

The total RNA was extracted with TRIzol reagent (Invitrogen), and cDNA was synthesized by PrimeScript™ RT reagent Kit with gDNA Eraser (TaKaRa #RR047A). SYBR® Premix Ex Taq™ GC (TaKaRa #RR071A) was used for RT-qPCR analysis. The primer sequences are listed in Table 1.

### 2.8. Lactate Assay and ELISA Assay

The assay medium for glycolytic capacity consisted of 2 mM glutamine in hippocampal XF basal medium [15]. The intracellular and extracellular concentrations of lactate were determined using the Lactate Colorimetric/Fluorometric Assay Kit (K607–100; BioVision) according to the manufacturer's instructions. The surface markers of M1 and M2 macrophages were determined by enzyme-linked immunosorbent assay kits, and the specific product numbers are as follows: TGF-*β* 1 (Abcam, ab119557), TNF alpha (Abcam, ab285327), CD163 (Abcam, ab272204), IL-1*β* (Beyotime, PI301), IL-10 (Beyotime PI522), IL-6 (Beyotime PI326), Arg1 (sangon biotech D721046), and iNOS (ab253219).

### 2.9. Statistical Analysis

Statistical analysis was performed using SPSS version 22.0 (IBM Corporation, New York, USA). Statistical significance was calculated by a two-tailed test. GraphPad Prism 8.0 (GraphPad Software, La Jolla, CA, USA) was applied to generate statistical analysis. Significance values are ^∗^*P* < 0.05, ^∗∗^*P* < 0.01, and ^∗∗∗^*P* < 0.001.

## 3. Results

### 3.1. Lactate Levels Are Elevated in Mice with Liver Fibrosis

To study the function of lactate in liver fibrosis, we first treated 8-week-old mice with a well-studied fibrosis inducer (CCl4) for 6 weeks. Then, liver fibrosis and liver morphology was assessed by hematoxylin and eosin (H&E) staining, Masson staining, and Sirius Red staining. H&E staining in the model group showed degeneration and necrosis of liver cells belonging to postnecrotic cirrhosis. Masson staining showed a large amount of blue collagen fiber deposition. The fiber cords were thick and stained deeply, indicating that there were many collagen fibers and had formed false lobules. Sirius Red staining showed that the collagen fibers of various types expanded outwards (Figure 1(a)). It turns out that the level of lactate is significantly higher in mice with liver fibrosis than in control mice (Figure 1(b)). As in previous study [17], we found that in fibrotic mice with elevated lactate, histone lactate levels were also significantly increased (Figure 1(c)). Alpha smooth muscle actin (*α*-SMA) is an indicator of HSC activation and a valuable marker of fibrosis progression and an early indicator of fibrosis development [27]. We detected the protein level of *α*-SMA by western blot and found that the protein level of *α*-SMA was indeed significantly increased in mice with liver fibrosis (Figure 1(d)). Importantly, elevated levels of acetylation in M1 macrophages promote their transformation into M2 macrophages [20]. So, we also used ELISA kit to detect the protein levels of M2 macrophage markers Arg1, CD163, and IL-10 and found that M2 macrophages in liver fibrosis mice were significantly higher than those in the control group, as in the previous study (Figure 1(e)) [10]. In conclusion, the levels of lactate, histone acetylation, and the number of M2 macrophages were significantly increased in liver fibrotic mice.

### 3.2. Activated HSC Cell Line LX-2 Can Stimulate the Transformation of M1 to M2 Macrophages

To explore the regulation of activated HSCs on the M1/M2 transformation of macrophages, we cultured LX-2 cells and treated them with TGF-*β* to obtain activated HSCs (aLX2). First, the increased level of *α*-SAM identified by western blot indicates that LX-2 is indeed activated (Figure 2(a)). In fact, consistent with previous findings, both glycolysis levels and lactate content were significantly increased in activated HSCs aLX-2 cells (Figures 2(b) and 2(c)). Then, the aLX-2 were cocultured with M1-type macrophages to observe whether M1 could transform into M2. We detected the following indicators by ELISA and found that the expression levels of M1 macrophage surface markers IL-1*β*, IL-6, iNOS, and TNF-*α* in co-aLX-2 cells and supernatants were markedly decreased, but the expression levels of M2 macrophage surface markers Arg1, CD163, IL-10, and TGF*β* were significantly increased (Figures 2(d) and 2(e)). Importantly, the level of histone acetylation was also significantly increased in co-LX-2 cells and their supernatants (Figure 2(f)). This suggests that activated HSCs aLX-2 can stimulate the transformation of M1 to M2 macrophages, which may be related to the accumulation of lactate and the promotion of histone acetylation.

### 3.3. Activated HSCs Can Stimulate the Transformation of M1 to M2 Macrophages

We previously demonstrated that activated LX-2 can stimulate the transformation of M1 to M2 macrophages in hepatic stellate cell lines, but it is unknown whether primary cell lines have the same function. So, we isolated and cultured HSCs from mice and used TGF-*β*1 to activate them. As shown in Figure 3(a), the protein level of *α*-SAM was significantly increased in activated HSCs compared with unactivated HSCs. Similarly, consistent with previous findings, both glycolysis levels and lactate content were significantly increased in activated HSCs (Figures 3(b) and 3(c)). Next, we examined the expression of M1 and M2 macrophage markers in the cell supernatants of cultured HSCs and activated HSCs and found that the expression levels of M1 macrophage surface markers IL-1*β*, IL-6, iNOS, and TNF-*α* in a-HSC supernatants were markedly decreased, but the expression levels of M2 macrophage surface markers Arg1, CD163, IL-10, and TGF*β* were significantly increased (Figures 3(d) and 3(e)). Importantly, the level of histone acetylation was also significantly increased in the supernatants of a-HSCs (Figure 3(f)). This suggests that activated primary HSCs can stimulate the transformation of M1 to M2 macrophages, which may be related to the accumulation of lactate and the promotion of histone acetylation.

### 3.4. Lactate Promotes the Transformation of M1 into M2 Macrophages by Promoting Histone Acetylation at the Promoters of Genes CD163, Arg-1, IL-10, and TGF-*β*1

To determine whether lactate can promote the conversion of M1 into M2 macrophages, we supplemented lactate in the medium in which M1 macrophages were cultured, and the results demonstrated that lactate indeed promoted the conversion of M1 into M2 macrophages (Figure 4(a)). To further analyze the mechanism of M1 into M2 macrophage transformation, we performed ChIP experiment with histone acetylation antibody. Since the level of histone acetylation in the promoter region of the M2 marker cannot be directly detected, we used histone acetylation antibody for ChIP experiment, and qPCR detected the expression of related genes. The higher the expression level of the genes, the higher the level of their histone acetylation. This also indicates that the higher level of histone acetylation bound to the promoter region of the M2 marker genes. Therefore, the levels of histone acetylation modifications at the promoter regions of genes (*Arg-1*, *CD*163, *IL-*10, and *TGF-β*1) were then examined by ChIP-qPCR. As shown in Figure 4(b), the levels of acetylation modification at the promoters of these genes were all significantly increased in M1 cells cultured with lactate. And immunoprecipitation assay showed that the acetylation of histone was mildly elevated in M2 macrophage transformed from M1 macrophage after treating with 20 mM lactate for 24 h (Figure 4(c)).

## 4. Discussion

Hepatic fibrosis is a major cause of morbidity and mortality worldwide because it ultimately leads to cirrhosis. Following liver injury, quiescent HSCs enter the cell cycle, differentiate, and maintain a chronic inflammatory response that accompanies fibrosis [28]. There is increasing evidence that hepatic fibrosis results in alterations in carbohydrate metabolism [12]. Glycolytic levels in both activated hepatic stellate cells and the entire fibrotic liver were significantly increased [29]. As the final product of the glycolytic pathway, whether lactate is important in hepatic fibrosis is particularly worth investigating. In our study, we first established a mouse model of liver fibrosis using CCl4 based on the previous research [30]. Considering that the cellular response to liver injury is highly dependent on sex [31], only female mice were used in our study. So, it was first demonstrated that both glycolysis levels and lactate were significantly increased in hepatic fibrotic mice (Figure 1). When liver injury occurs, HSCs are activated and generate an extracellular matrix network, resulting in the appearance of fibrotic scars [32]. Importantly, it was also shown that the level of lactate was significantly increased in both activated HSC cell line and activated primary HSCs in this study (Figures 2 and 3).

The mechanisms linking M1/M2 macrophage transformation to the development of hepatic fibrosis remain a subject of intensive research, highlighting the necessity to better understand the complex functional interactions that occur between the two macrophage types in the liver [33]. Extracellular signals from activated HSCs, macrophages, and hepatocytes are thought to be essential mediators of the fibrotic cascade in hepatic fibrosis [34, 35]. A previous research shows that phenotypic switching between M1 and M2 can occur under specific stimuli in vivo and in vitro [14]. Interestingly, the number of hepatic M2 macrophages is positively correlated with the severity of liver fibrosis [10]. Considering that the elevated level of lactate modification in M1 macrophages can promote the transformation of macrophages into M2 macrophages [20], we detected the surface markers (Arg-1, CD163, IL-10, and TGF-*β*1) of M2 macrophages after adding lactate to the culture medium when culturing M1 macrophages. The results demonstrated that lactate indeed promoted the conversion of M1 into M2 macrophages (Figure 4). With ChIP-qPCR assay, we found that the levels of acetylation modification at the promoters of these genes were all significantly increased in M1 cells cultured with lactate. However, this study only describes the phenomenon of M1 and M2 conversion and the effect of lactate and histone acetylation on the conversion of M1 to M2, and the molecular mechanism has not been elucidated, which needs to be further studied.

In conclusion, we demonstrate that activated HSCs can promote the progression of liver fibrosis by secreting a large amount of lactate, increasing the level of histone lactate modification in hepatic M1 macrophages, and promoting the transformation of M1 into M2 macrophages (Figure 5). This fact provides us with new insights into the generation of liver fibrosis and provides an optimistic view that lactate inhibitors or acetylation inhibitors may be used in the treatment of liver fibrosis and reducing the incidence of liver cancer. Overall, modulation of HSCs can prevent and treat liver fibrosis by inhibiting the activation of HSCs, promoting the phenotypic transformation of HSCs, promoting apoptosis of HSCs, and inducing senescence of HSCs. Currently, one of the main focuses of fibrosis research is the development of targeted therapies with high liver specificity. Therefore, further investigation of the mechanisms involved in HSC activation may provide new therapeutic targets for the treatment of liver fibrosis.

## Figures and Tables

**Figure 1:** Lactate levels are elevated in mice with liver fibrosis. (a) The 8-week-old mice were treated with CCl4 for 6 weeks, and the fibrosis was assessed by H&E, Masson, and Sirius red staining. Scale bars are 100 *μ*m. (b) Kit to detect lactate level in the liver tissue. At least 3 liver sections were analyzed per mouse (number of mice: *n* = 12). (c, d) Western blot showing expression of acetylation and *α*-SMA in the livers of mice treated with CCl4. (e) Detection of the expression levels of M2 macrophage surface markers CD163, Arg1, and IL-10 in the liver by ELISA. ^∗∗^*P* < 0.01, ^∗∗∗^*P* < 0.001.

**Figure 2:** HSCs regulate the transformation of M1/M2 macrophages. (a) Western blot showing expression of *α*-SMA in the aLX-2. Activated HSCs (aLX-2) were obtained by treating LX-2 cells with TGF-*β*. (b) Lactate level in aLX-2. (c) The level of glycolysis in aLX-2. (d) Detection of the expression levels of M1 macrophage surface markers IL-1*β*, IL-6, iNOS, and TNF-*α* in transformed THP-1 cells cultured with aLX or its supernatant and their supernatants by ELISA. (e) Detection of the expression levels of M2 macrophage surface markers Arg1, CD163, IL-10, and TGF*β* in co-aLX-2 co-LX-a cells and their supernatants by ELISA. (f) Western blot showing expression of acetylation n co-aLX-2 co-LX-a cells and their supernatants. ^∗^*P* < 0.05, ^∗∗^*P* < 0.01, and ^∗∗∗^*P* < 0.001.

**Figure 3:** Regulation of primary activated HSCs on the M1/M2 phenotypic transition of macrophages. (a) Western blot showing expression of *α*-SMA in the HSC and a-HSC (activated HSCs). (b) Lactate level in HSCs and a-HSCs. (c) The level of glycolysis in HSCs and a-HSCs. (d) Detection of the expression levels of M1 macrophage surface markers IL-1*β*, IL-6, iNOS, and TNF-*α* in co-aLX-2 co-LX-a cells and their supernatants by ELISA. (e) Detection of the expression levels of M2 macrophage surface markers Arg1, CD163, IL-10, and TGF*β* in the supernatants of HSCs and a-HSCs by ELISA. (f) Western blot shows the expression of histone acetylation in the supernatants of HSCs and a-HSCs. ^∗^*P* < 0.05, ^∗∗^*P* < 0.01, and ^∗∗∗^*P* < 0.001.

**Figure 4:** Lactic acid stimulates the conversion of M1 to M2 macrophages. (a) The mRNA expression levels of Arg-1, CD163, IL-10, and TGF-*β*1 in M1 macrophages cultured with and without lactate by qPCR. (b) The levels of histone acetylation modifications at the promoter regions of genes (Arg-1, CD163, IL-10, and TGF-*β*1) were examined by ChIP-qPCR. (c) IP-western blot detected the level of histone acetylation inM1 macrophages after treated with 20 mM lactate or vehicle for 24H. ^∗^*P* < 0.05, ^∗∗^*P* < 0.01, and ^∗∗∗^*P* < 0.001.

**Figure 5:** Schematic representation of the process that activated HSCs promoted M1 to M2 macrophage transformation and liver fibrosis by elevating the histone acetylation level.

**Table 1:** Real-time PCR primer sequences.

Gene	Sense (5′-3′)	Antisense (5′-3′)
CD163	TCAGCTGATTTCAGTGCTGCT	TCACGTAACTGTGAGGCTCTT
Arg1	TGACTGAAGTAGACAAGCTGGGGAT	CGACATCAAAGCTCAGGTGAATCGG
IL-10	GAAAGGAAGCCAGCTACCCC	ACAGAATCTCCCCGTTAGCC
TGF-*β*1	GGCAATCTACAAGTTCATTGGGC	AAGGAACCGCAGCACTCATA

## Data Availability

The data used to support the findings of this study are included within the manuscript.

## References

[1] Kisseleva T., Brenner D. (2021). Molecular and cellular mechanisms of liver fibrosis and its regression. *Nature Reviews Gastroenterology & Hepatology*.

[2] Dhar D., Baglieri J., Kisseleva T., Brenner D. A. (2020). Mechanisms of liver fibrosis and its role in liver cancer. *Experimental Biology and Medicine*.

[3] Friedman S. L. (2003). Liver fibrosis – from bench to bedside. *Journal of Hepatology*.

[4] Lo R. C., Kim H. (2017). Histopathological evaluation of liver fibrosis and cirrhosis regression. *Clinical and Molecular Hepatology*.

[5] Khomich O., Ivanov A. V., Bartosch B. (2020). Metabolic hallmarks of hepatic stellate cells in liver fibrosis. *Cells*.

[6] Geerts A. (2001). History, heterogeneity, developmental biology, and functions of quiescent hepatic stellate cells. *Seminars in Liver Disease*.

[7] Senoo H., Kojima N., Sato M. (2007). Vitamin A-storing cells (stellate cells). *Vitamin A*.

[8] Hazra S., Xiong S., Wang J. (2004). Peroxisome proliferator-activated receptor *γ* induces a phenotypic switch from activated to quiescent hepatic stellate cells.

[9] Koyama Y., Wang P., Liang S. (2017). Mesothelin/mucin 16 signaling in activated portal fibroblasts regulates cholestatic liver fibrosis. *Journal of Clinical Investigation*.

[10] Xi S. J., Zheng X., Li X. (2021). Activated hepatic stellate cells induce infiltration and formation of CD163^+^ macrophages *via* CCL2/CCR2 pathway. *Frontiers in Medicine*.

[11] Iredale J., Campana L. (2017). Regression of liver fibrosis. *Seminars in Liver Disease*.

[12] Shi X., Shi L., Zhang S. (2020). Mechanistic study of vitamin C attenuation of endometriotic fibrosis. *Clinical and Experimental Obstetrics & Gynecology*.

[13] Xue Y., Nie D., Wang L. J. (2021). Microglial polarization: novel therapeutic strategy against ischemic stroke. *Aging and Disease*.

[14] Sica A., Invernizzi P., Mantovani A. J. H. (2014). Macrophage plasticity and polarization in liver homeostasis and pathology. *Hepatology*.

[15] Alves-Bezerra M., Cohen D. E. (2017). Triglyceride metabolism in the liver. *Comprehensive Physiology*.

[16] Wang W., Wang C., Xu H., Gao Y. (2020). Aldehyde dehydrogenase, liver disease and cancer. *International Journal of Biological Sciences*.

[17] Zhang D. (2019). Metabolic regulation of gene expression by histone lactylation. *Nature*.

[18] Lu Z., Li X., Yang P. (2021). Heparin-binding protein enhances NF-*κ*B pathway-mediated inflammatory gene transcription in M1 macrophages via lactate. *Inflammation*.

[19] Smith-Cortinez N., van Eunen K., Heegsma J. (2020). Simultaneous induction of glycolysis and oxidative phosphorylation during activation of hepatic stellate cells reveals novel mitochondrial targets to treat liver fibrosis. *Cell*.

[20] Irizarry-Caro R. A., McDaniel M. M., Overcast G. R., Jain V. G., Troutman T. D., Pasare C. (2020). TLR signaling adapter BCAP regulates inflammatory to reparatory macrophage transition by promoting histone lactylation. *Proceedings of the National Academy of Sciences of the United States of America*.

[21] Zhao C., Dong H., Xu Q., Zhang Y. (2020). Histone deacetylase (HDAC) inhibitors in cancer: a patent review (2017-present). *Expert Opinion on Therapeutic Patents*.

[22] Yang J. J., Yang Y., Zhang C., Li J., Yang Y. (2020). Epigenetic silencing of lncRNA ANRIL enhances liver fibrosis and HSC activation through activating AMPK pathway. *Journal of Cellular and Molecular Medicine*.

[23] Sayed N., Khurana A., Saifi M. A., Singh M., Godugu C. (2019). Withaferin a reverses bile duct ligation-induced liver fibrosis by modulating extracellular matrix deposition: role of LOXL2/Snail1, vimentin, and NF*κ*B signaling. *BioFactors*.

[24] You D. G., Oh B. H., Nguyen V. Q. (2021). Vitamin A-coupled stem cell-derived extracellular vesicles regulate the fibrotic cascade by targeting activated hepatic stellate cells in vivo. *Journal of Controlled Release*.

[25] Geerts A., Eliasson C., Niki T., Wielant A., Vaeyens F., Pekny M. (2001). Formation of normal desmin intermediate filaments in mouse hepatic stellate cells requires vimentin. *Hepatology*.

[26] Lan F., Collins R. E., de Cegli R. (2007). Recognition of unmethylated histone H3 lysine 4 links BHC80 to LSD1-mediated gene repression. *Nature*.

[27] Akpolat N., Yahsi S., Godekmerdan A., Yalniz M., Demirbag K. (2005). The value of alpha-SMA in the evaluation of hepatic fibrosis severity in hepatitis B infection and cirrhosis development: a histopathological and immunohistochemical study.

[28] Zhang D. Y., Friedman S. L. J. H. (2012). Fibrosis-dependent mechanisms of hepatocarcinogenesis. *Hepatology*.

[29] Chang M.-L., Yang S.-S. J. C. (2019). Metabolic signature of hepatic fibrosis: from individual pathways to systems biology. *Cells*.

[30] Yang W., He H., Wang T. (2021). Single-cell transcriptomic analysis reveals a hepatic stellate cell–activation roadmap and myofibroblast origin during liver fibrosis in mice. *Hepatology*.

[31] Naugler W. E., Sakurai T., Kim S. (2007). Gender disparity in liver cancer due to sex differences in MyD88-dependent IL-6 production.

[32] Bataller R., Brenner D. A. (2005). Liver fibrosis. *The Journal of clinical investigation*.

[33] Rahman N., Pervin M., Kuramochi M. (2018). M1/M2-macrophage polarization-based hepatotoxicity in d-galactosamine-induced acute liver injury in rats. *Toxicologic Pathology*.

[34] Friedman S. L. J. G. (2008). Mechanisms of hepatic fibrogenesis. *Gastroenterology*.

[35] Thomas J. A., Pope C., Wojtacha D. (2011). Macrophage therapy for murine liver fibrosis recruits host effector cells improving fibrosis, regeneration, and function.

